RETRACTED

# Dermoscopic and reflectance confocal microscopic features of children scabies

**DOI:** 10.1111/srt.13459

**Published:** 2023-09-07

**Authors:** Zhiwei Guan, Tiantian Bi, Qinfeng Li

**Affiliations:** ^1^ Department of Dermatology Tianjin Children's Hospital Tianjin China

**Keywords:** children, dermoscopy, reflectance confocal microscopy, scabies

## Abstract

**Objective:**

To summarize the image features of dermatoscopy and reflectance confocal microscopy (RCM) in children with scabies, and to explore the clinical significance in the diagnosis of children scabies.

**Methods:**

A retrospective analysis was conducted on 102 children scabies diagnosed clinically in the dermatology outpatient department of Tianjin Children's Hospital from April 2018 to June 2022. All children were examined by dermatoscopy and RCM, and images were collected.

**Results:**

102 patients, 92 patients (90.2%) showed characteristic dermoscopic manifestations: white tunnels and small brown or dark brown triangular structures at their ends. 91 patients (89.2%) showed characteristic reflectance confocal microscopic manifestations: tunnels, scabies mites, feces, and eggs in the epidermal layer. All patients showed different degrees of non‐specific manifestations of dermoscopy and RCM.

**Conclusion:**

Children scabies have typical dermatoscopic and reflectance confocal microscopic characteristics, and dermatoscopy and RCM are effective non‐invasive diagnostic methods with high clinical application value in the diagnosis and differential diagnosis of children scabies.

## 1 INTRODUCTION

Scabies is a highly infectious skin parasitic disease caused by scabies mites. The misdiagnosis rate is high in clinical practice. Early detection and timely treatment are essential. The form and distribution of scabies rash in children are often atypical, and there are few studies on dermoscopy and RCM. The current literature is mainly case reports. By summarizing the image characteristics of children scabies under dermatoscopy and RCM, this paper provides a non‐invasive, diagnostic, differential diagnosis and follow‐up method after treatment for children scabies.

## 2 MATERIALS AND METHODS

### 2.1 Patients

A retrospective analysis was conducted on 102 patients diagnosed with scabies in the dermatology department of Tianjin Children's Hospital from April 2018 to June 2022.

### 2.2 Diagnostic criteria

The 2020 IACS standard includes three levels: A. Confirmed scabies (meeting at least one of the following three criteria) A1: Skin lesions were taken and observed under an optical microscope with scabies, insect eggs, or feces; A2: Scabies mites, insect eggs, or feces visible under high‐power imaging system; A3: Dermatoscopy revealed scabies mites. B. Clinical diagnosis of scabies (meeting at least one of the following three criteria) B1: scabies tunnel; B2 typical skin lesions involving male genital areas; B3: There are typical skin lesions in typical areas, plus two medical history features. C: Suspected scabies (two in line with one) C1: There is a typical skin lesion in a typical area, plus one medical history feature; C2: Atypical site or skin lesion, plus two medical history features. H. Medical history characteristic H1: itching; H2 positive contact history. Diagnosis can be at one of three levels (A, B, or C).^1^

RETRACTED

### 2.3 Instrument

The Dermoscope‐ II desktop of Beijing Demetricom was used to observe 102 children. The lens is in parallel contact with the skin lesion, and 75% ethanol is used as the infiltrating liquid.

RCM (vivascope3000) is produced by Lucid Corporation in the United States. The light source is a laser beam with a wavelength of 830 nm, with a maximum output of 16 mw and a lateral resolution of 0.5–1.0 μm. Axial resolution of 3–5 μm. The lens is a ×30 water immersion objective with a magnification of ×40–100.

Adjust the best angle and image definition, and collect the dermoscopic and RCM images of the skin lesion. All images were collected by the same staff.

### 2.4 Examination method

Select multiple skin lesions for scanning, and refer to the literature for the examination method; Select the prone areas for skin lesions: external genitalia, interphalanges, and armpits. Detected positive for scabies, mites, or eggs.

## 3 RESULTS

### 3.1 Clinical characteristics of children scabies

A total of 102 patients: 59 males (57.8%) and 43 females (42.2%), aged 0–14 years old, with the youngest patient being 1 month old. The average age is 4.08 ± 4.06 years old.

Rash characteristics: The primary lesions are erythema, papules, blisters, papules, nodules, and tunnels, while secondary lesions include scabs, erosion, exudates, pustules, scales, and pigmentation. Paules, papules, nodules, and tunnels are mostly edematous red and non‐edematous brown in color. The rash on the palms and soles shows blisters, bullae, and pustules (Figure 1).

**FIGURE 1:** Clinical characteristics of children scabies. (A) Red papules and papulovesicles can be seen between the fingers, and blisters can be seen on the back of the fingers. (B) Red papules and nodules can be seen under the armpit. (C) Red nodules can be seen on the penis, and white tunnels can be seen on the surface of the nodules. (D) Erythema, papules, nodules, scratches, ulcers, and scabs can be seen on the buttocks.

### 3.2 Dermatoscopic features

The positive rate is 90.2% (92/102).

RETRACTED

The characteristic dermoscopic manifestations of scabies: A white tunnel and its brown or dark brown small triangular structure at the end (Figure 2).

**FIGURE 2:** The characteristic dermoscopic manifestations. (A) Short wide groove shaped tunnel. (B) Thin long groove shaped tunnel. (C) Shallow desquamation linear tunnel and insect eggs. The tunnel is a cave, and the dark triangular structure is the body of scabies mites. (D) The gray black lines (black arrows) visible at the edge of the tunnel in the picture represent feces containing melanin. (E) multiple scabies mites' structures visible at the same time (black arrow).

The non‐characteristic dermoscopic manifestations of scabies: Mainly secondary skin lesions caused by itching, such as erythema, pustules, erosion, exudation, scratches, blood scabs, pigmentation, vascular changes, and so forth (Figure 3).

**FIGURE 3:** The non‐characteristic dermoscopic manifestations. (A) collar shaped desquamation, as a pseudo tunnel. (B) scratches, scabbing, and ulceration. (C) multiple dry blisters and pustules, with a tunnel and inverted triangular structure visible in the upper right corner. (D) collar shaped desquamation, with a cluster of dotted vascular structures visible in the center. (E) Y‐shaped trajectory, with multiple dry blister structures visible in the trajectory area, and yellow white scabs visible around it. (F) pigmentation, white patches, and focal spherical vascular structures.

### 3.3 RCM features

The positive rate is 89.2% (91/102).

The non‐characteristic RCM manifestations of scabies: Compared to the surrounding normal skin, varying degrees of edema can be observed in the epidermis and dermis of the lesion area, with blister formation visible, unclear boundaries of the dermis, diffuse infiltration of inflammatory cells, and aggregation of neutrophils to form pustules (Figure 4A,B).

**FIGURE 4:** RCM features. (A) Epidermal edema, blister formation. (B) Diffuse infiltration of inflammatory cells and aggregation of neutrophils to form pustules. (C) Medium to high refractive tunnel structure, with an opening on the epidermis (red arrow), a cavity (white arrow) as the tunnel entrance, and an elliptical insect egg (blue arrow). (D) Typical tunnels before treatment. (E) The head and forelimbs of the scabies (orange arrows), and multiple oval high refractive index structures arranged in a linear pattern, consisting of scabies mite feces (yellow arrow) and containing the eggs of the mite embryo (blue arrows). (F) Clear boundary of scabies mite body, visible head and two pairs of forelegs (orange arrows). (G) Oval, well‐defined insect eggs (blue arrow), circular strongly refracted feces (yellow arrow). (I) After three days of treatment, the head and forelimbs of the scabies mite can still be seen (orange arrow), but the oval high refractive fecal particles and eggs containing embryos disappear (the same skin lesion as C). (J) After three days of treatment, the original tunnel narrowed and a small amount of highly refractive irregular clumps were visible inside (the same skin lesion as D).

RETRACTED

The characteristic RCM manifestations of scabies: Visible tunnels, mites, feces, and eggs (Figure 4C–J).

## 4 DISCUSSION

Scabies is a contagious skin disease caused by the parasitism of scabies mites within the epidermal layer of the human skin. Scabies mites often parasitize in thin and tender areas of the skin, such as fingertips, wrist flexion, umbilical fossa, groin, scrotum, and external genitalia.^2^ The stratum corneum of children is thin, the form and distribution of scabies rash is not typical, and non‐prone parts, including the scalp, face, palm, and sole, can develop rashes,^3^ often confused with eczema dermatitis, prurigo nodosa, Langerhans histiocytosis, acral pustulosis, papular Hives, prickly heat, pigmented Hives, and so forth.^4^, ^5^ Some younger children are unable to express, so childhood scabies are easily misdiagnosed. The direct microscopic examination or biopsy of scabies mites and their eggs or feces is the gold standard for diagnosing scabies.^6^, ^7^ However, experimental sampling often causes damage to the insect body, eggs, and fecal particles due to the scraping process, and the detection amount of intact insect bodies, eggs, and fecal particles is not high.^8^ The sampling process can cause discomfort to patients and cannot be well coordinated. Therefore, there are many limitations in the diagnosis of scabies by traditional auxiliary means. Reflective confocal microscope (RCM) and dermoscope are new skin imaging diagnostic technology, that have demonstrated improved efficacy in the diagnosis of scabies.^9^, ^10^, ^11^

The typical dermoscopic manifestation of scabies is a white tunnel with a brown or dark brown small triangular structure at its end. The white tunnel has irregular wavy lines and is excavated by female mites to lay eggs, containing insect eggs and fecal balls. The brown small triangle structure is composed of the head and two pairs of forelegs of the scabies mite. Similar to Jet aircraft or triangle gliders. The triangular glider and the wake represent the mouth and cave of the scabies mite, respectively.^12^, ^13^, ^14^ Sarcoptes parasitizes in the deep Stratum corneum of the host epidermis, feeds on the cuticle tissue and lymph, and digs with the pincers and the front tarsal claw, gradually forming a winding tunnel parallel to the skin, with the longest tunnel dug by the female mite.^3^, ^15^, ^16^ The length of the tunnel can indicate the activity of scabies mites, and the short and wide trench‐shaped tunnel may indicate that this is a male mite. The circular trajectory around it suggests that it may be caused by the crawling of female mites that have completed fertilization; The slender groove‐like tunnel suggests that it may be a pre‐fertilization female mite; Shallow shedding linear tunnels and insect eggs indicate the presence of fertilized female mites here, which are most susceptible to infection with new hosts during this period.^17^ This study also found that under the skin microscope, large areas of collar‐like desquamation were visible in some children, showing a tunnel‐like appearance, indicating that there may have been active crawling mites here. The grayish‐black lines at the edge of the tunnel may be caused by scabies mite phagocytosis of Keratinocyte containing melanin, which is concentrated and released in the form of feces, then arranged in a curve and adhered to each other.^18^ In this study, 102 patients underwent dermoscopic examination, of which 92 patients showed characteristic manifestations, and the sensitivity for diagnosing scabies was 90.2%, similar to literature reports.^19^, ^20^ Ten patients did not exhibit characteristic manifestations, possibly due to erosion, scratches, and blood scabs covering or masking the primary lesion. Surprisingly, out of these 10 patients, seven underwent RCM examination and found worm bodies and eggs. The combined examination improved the positive rate of diagnosis. The dermoscopic features of scabies summarized in this study clearly demonstrate the parasitic state of scabies, providing a more intuitive understanding of scabies. Dermoscopy can effectively reduce the misdiagnosis rate of clinical physicians. In addition, this study also found that non‐characteristic manifestations of dermoscopy were overlooked in previous studies. The significance of non‐specific structures lies in discovering atypical scabies or suggesting complex infections and allergic states in different patients, as well as varying degrees of skin barrier damage.

RETRACTED

RCM is a real‐time, dynamic, non‐invasive skin detection device that can observe tunnels, mites, eggs, and feces in real‐time in the body.^21^ In these microscopic features, it is highly specific to find scabies mites, scabies eggs, or dung ball structures for the diagnosis of scabies, and scabies can be diagnosed when one of the three is found under RCM, dung ball is the most common feature of reflex confocal microscope in scabies, and its sensitivity and specificity are high. It is of great significance to diagnose scabies.^22^, ^23^ In this study, 102 patients underwent RCM examination, of which 91 patients showed characteristic manifestations, with a sensitivity of 89.2% for the diagnosis of scabies, which is similar to literature reports.^24^ The remaining 11 cases showed no appearance of scabies mites, which were considered to be related to scratching stimulation, damage to the skin, scab debris covering the structure of scabies mites, longer examination time, slightly poor cooperation of the patient, or fewer sampling sites. RCM can observe the movement of scabies mites, monitor their survival in the body, and help determine the efficacy of anti‐scabies drugs in clinical practice.^25^ Traditionally, observing the movement of scabies mites under an optical microscope after scraping the skin is considered the only way to confirm their survival ability in laboratory environments. However, the lack of movement observed under an in vitro optical microscope by scabies mites is not a reliable indicator of insecticide efficacy, as this may be caused by traumatic damage to parasites during the scraping process. RCM can be non‐invasive and clearly observe the activity of parasites before and after treatment.^26^ In this study, RCM showed that before treatment, insect eggs and more highly refractive fecal particles were visible around the scabies mites. After treatment, although the clinical skin lesions did not subside significantly, RCM showed no feces or insect eggs around the same site of the scabies mites. The quantity of insect eggs and feces can to some extent reflect the survival activity of scabies mites, indicating that although the skin lesions subside slowly, anti‐scabies treatment is effective; After continuing treatment, follow‐up examination showed that both the body and eggs of the scabies mites disappeared. Based on the patient's skin lesions and RCM examination results, medication discontinuation can be guided. Therefore, conducting RCM examination in suspicious areas is very helpful in confirming the presence of scabies mites and determining their survival after treatment. In addition, the non‐specific manifestations of RCM, as well as the strong inflammatory response in the true epidermis, also have a certain suggestive effect on parasitic infection.

The observation content of dermoscopy is a superimposed image from the surface of the skin lesion to the superficial dermis in a vertical direction, while the observation content of RCM is the cell level at any section from the epidermis to the dermis. The skin lesions magnified under dermoscopy can accurately reflect the subtle changes in the lesions, but cannot be identified at the cellular level. Low magnification rates cannot observe eggs and feces. In addition, for inexperienced examiners, the so‐called “brown small triangular structure” is prone to mixing with scabs, dander, small dust particles, and so forth. In addition, areas with more hair are not conducive to dermoscopic observation, and its application in the diagnosis of scabies has certain limitations. However, the dermoscopy is simple in operation, which can quickly find tunnel structures or inverted triangular structures, facilitating the location of skin lesions. RCM is not as intuitive and sensitive as dermoscopy in terms of changes in the surface of skin lesions, but RCM is more specific in terms of inspection of scabies mite bodies, eggs, and feces. The combination of dermoscopy and RCM can increase the positive rate of scabies diagnosis.

RETRACTED

## CONFLICT OF INTEREST STATEMENT

The authors declare that the research was conducted in the absence of any commercial or financial relationships that could be construed as a potential conflict of interest.

## Data Availability

Data were derived from public resources.
